This article has been retracted.

# Effect of Immediate Breast Reconstruction after Standardized Breast Cancer Surgery on the Quality of Life of Patients: A Prospective Multicenter Study

**DOI:** 10.1155/2021/2840043

**Published:** 2021-10-26

**Authors:** Chao Zhang, Hongchuang Jiang

**Affiliations:** Department of Breast Surgery, Beijing Chao-Yang Hospital, Capital Medical University, Beijing 100020, China

## Abstract

**Objective:**

To investigate the impact of immediate breast reconstruction (IBR) after standardized breast cancer (BC) surgery on the quality of life of patients.

**Methods:**

A total of 878 BC patients were included, who were diagnosed and treated in the breast surgery department between January 2016 and December 2018. The patient underwent immediate postoperative breast reconstruction surgery. Subsequently, safety, efficacy, and postoperative morphology were scored and evaluated for the comprehensive analysis of the clinical therapeutic effects.

**Results:**

With longer postoperative time, a lower proportion of the follow-up population experienced limb edema, capsular contracture, infection, calcifications around the prosthesis, prosthesis dislocation, delayed wound healing, chronic lymphadenopathy, pain, and prosthesis rupture, indicating a high safety. And the follow-up patients' breast appearance and shape largely returned to normal at 12 months postoperatively. Additionally, patients with 3 and 6 months of follow-up had a higher quality of life and better aesthetic breast reconstruction outcomes compared to the perioperative period.

**Conclusion:**

The implementation of standardized IBR after breast cancer improves the quality of life of patients after surgery with fewer complications and a good safety profile.

## 1. Introduction

Breast cancer (BC) has the highest incidence among tumors in females, especially in women in the Asia-Pacific region where BC accounts for 18% of all cases [1]. Radical mastectomy is the first choice for the treatment of BC [2], but postoperative patients are often unable to face reality during rehabilitation. Specifically, postoperative patients have avoidance behaviors such as reducing social activities, communication disorders, and avoiding physical contact [3], which negatively affect the patient's mood, psychology, self-aesthetics, and social life [2]. Surgery is the mainstay of treatment for BC and is diverse, including reconstructive surgery. In recent years, with the rapid development of China's economy and the continuous improvement of people's living standards, in addition to the purpose of continuing life, the quality of life of patients has also received much attention in BC treatment [4]. Therefore, breast reconstruction has become popular, generally including immediate breast reconstruction (IBR) and delayed breast reconstruction (DBR). Some studies have suggested that IBR is superior to DBR in reducing the number of operations and the risk of surgery and shortening postoperative recovery time. Additionally, IBR has lower cost and higher patient satisfaction, effectively improving the quality of life of patients [5–7]. In this study, with BC patients as the study subjects, safety, efficacy, and postoperative morphology of IBR are evaluated through comparative analysis, and subsequently, the effect of IBR on the quality of life of BC patients is investigated.

## 2. Materials and Methods

### 2.1. Inclusion and Exclusion Criteria

This study is a prospective, multicenter trial. The trial procedures were performed in accordance with the relevant institutional, national, and international guidelines and regulations and were approved by the Medical Ethics Committee of Beijing Chaoyang Hospital, Capital Medical University (2016-4-29-1). BC patients diagnosed and treated in the breast surgery department of multiple tertiary hospitals between January 2016 and December 2018 were collected. A total of 878 patients were included in this study.

The inclusion criteria were as follows: (1) age ≥18 years; (2) patients were diagnosed as BC by pathological examination; (3) no previous BC treatment; (4) patients underwent IBR after BC surgery; (5) no breast tissue inflammation, obvious infection in other parts, or no inflammatory BC; (6) patients without the tendency of recurrence of metastasis of residual tumor after BC surgery; (7) body mass index (BMI) < 30; (8) patients voluntarily signed informed consent.

The exclusion criteria were as follows: (1) patients underwent DBR after BC surgery; (2) patients with severe lesions of the heart, lung, liver, kidney, and other important organs and malignant tumors in other parts; (3) patients with allergic diathesis, scar diathesis, and other systemic conditions that cannot tolerate breast plastic surgery; (4) pregnant or lactating patients; (5) patients with other immunological, physiological abnormal reactions; (6) patients who require postoperative adjuvant radiotherapy; (7) patients with regular smoking history; (8) patients with poor compliance who cannot cooperate to complete postoperative routine treatment and follow-up; (9) patients with psychological disorders or mental disorders.

### 2.2. Operation Procedures

Breast reconstruction was performed immediately after mastectomy. (1) Modified radical mastectomy (SSM)/nipple-areola-complex sparing mastectomy (NSM); (2) sentinel lymph node biopsy (SLNB)/axillary lymph node dissection (ALND); (3) breast reconstruction: 1. application of prosthesis/prosthesis + patch [8]; 2. application of the expander; 3. latissimus dorsi combined with prosthesis; 4. latissimus dorsi myocutaneous flap; 5. rectus abdominis myocutaneous flap (mainly transverse rectus abdominis myocutaneous flap) [9]; 6. deep inferior epigastric artery perforator flap [10].

### 2.3. Breast Measurements

According to the method described by Wang et al. [11], the following indicators were measured, including breast base diameter (width), breast height, breast protrusion, breast volume, and subcutaneous soft tissue thickness. The prosthesis was selected according to the values of the first three indicators in combination with the prosthesis standards of various manufacturers and the patient's requirements for postoperative breast shape.

### 2.4. Outcome Measures

The quality of life of patients in the two groups was observed after clinical treatment and was evaluated by the Chinese version of Functional Assessment of Cancer Therapy-Breast (FACT-B). The scale includes items of physical status, functional status, social/family status, emotional status, and additional concerns, and the higher the score, the better the quality of life of patients.

### 2.5. Efficacy Evaluation

Safety: capsular contracture, infection, calcifications around the prosthesis, prosthetic dislocation (exposure) and ruptures, delayed wound healing, chronic lymphadenopathy, pain, and autoimmune complications.

Effectiveness: standard chest circumference, breast type, breast position, skin texture, skin sensation, breast appearance, nipple morphology, and overall postoperative feeling. The postoperative morphology score is determined based on the breast appearance, flexibility, symmetry, subjective feeling, and overall satisfaction. The satisfaction of IBR after mastectomy was evaluated subjectively by both the surgeon and the patient, and the aesthetics of the reconstructed breast was assessed using Harris evaluation criteria [12].

### 2.6. Statistical Analysis

All experimental data were statistically analyzed using SPSS 22.0. Two-sample *T*-test was adopted for comparing the means of the two groups, and the enumeration data were analyzed by *χ*^2^ test. The results were expressed as mean ± standard deviation (SD), and *P* < 0.05 indicated a statistically significant difference.

## 3. Results

### 3.1. Clinical Baseline Characteristics

The baseline characteristics of the patients (Table 1) were as follows: age: about 46.28 ± 9.43 years; BMI: about 22.62 ± 3.87; income: <5000 yuan (*n* = 294), 5000–10000 yuan (*n* = 352), or >10000 yuan (*n* = 111); marital status: divorced (*n* = 16), married (*n* = 99), and unmarried (*n* = 754). A total of 192 patients had given birth, with 2.23 times of pregnancies, 1.29 times of deliveries, and about 9.66 months of lactation. Additionally, 104 cases were menopause women, 17 cases with hypertension and 3 cases with diabetes.

The tumor conditions of the patients were as follows: tumor location: upper-inner quadrant (*n* = 74), lower-inner quadrant (*n* = 21), upper-outer quadrant (*n* = 246), lower-outer quadrant (*n* = 53), and central area (*n* = 45); tumor size: about 2.24 ± 1.64 cm; tumor metastasis: no distal metastasis (*n* = 402) and distal metastasis (*n* = 24); histopathological grade: nonassessable (*n* = 89), low (*n* = 70), medium (*n* = 146), and high (*n* = 58); pathological diagnosis: invasive carcinoma (*n* = 333), carcinoma in situ (*n* = 78), and others (*n* = 24).

### 3.2. Postoperative Outcomes of Patients

The postoperative outcomes of the patients (Table 2) were as follows: postoperative chemotherapy: *n* = 211 (50.48%); number of drainage tubes: 1 (*n* = 5), 2 (*n* = 395), 3 (*n* = 28), and 4 (*n* = 4); IBR: *n* = 865 (98.52%); psychological status of patients at admission: any one or more of anxiety, irritability, and fear (*n* = 318) and normal (*n* = 95); acceptance of physical changes at discharge: acceptable (*n* = 23) and unacceptable (*n* = 442); total hospital stay: about 16 days; total cost: about 12823 yuan; number of recurrences: *n* = 4 (0.83%); metastasis: *n* = 8 (1.67%).

### 3.3. Postoperative Safety Assessment

Subsequently, we evaluated the patients for postoperative complications (Table 3). At 1 month after operation, the number of patients with breast infection (*n* = 13) and prosthesis rupture (*n* = 16) was higher than that of other indicators. However, at 3 months after operation, the number of patients with edema of the affected limb, capsular contracture, calcifications around the prosthesis, breast atrophy and thoracic deformity, and chronic lymphadenopathy began to increase. At 6 months after operation, there was one patient with calcifications around the prosthesis and one case of delayed wound healing. At 12 months after operation, none of the above conditions occurred.

### 3.4. Status of the Reconstructed Breast in Patients Followed Up at 3, 6, and 12 Months after Operation

The results of the follow-up showed that only 9 patients had tense and elastic breast skin texture at 3 months after surgery, but 63 patients had normal breast appearance, and 77 patients had normal nipple shape and size. At 6 and 12 months after surgery, only 3 patients had asymmetrical breast shape on both sides, and all other patients had normalized their breast condition (Table 4).

### 3.5. FACT-B Scores of Patients in the Perioperative Period and at 3 and 6 Months after Operation

The results of FACT-B scores showed that patients had lower FACT-B scores at both 3 and 6 months after operation than those in the perioperative period (*P* < 0.01). And the FACT-B scores were higher at 6 months after surgery compared with 3 months after surgery, but there was no significant difference (*P* > 0.05) (Figure 1).

### 3.6. Postoperative Breast Aesthetics in the Perioperative Period and at 3 and 6 Months after Operation

Breast aesthetic evaluation by the Harris scale (excellent, good, fair, and poor) showed that, in the perioperative period, there were 38.18% of the patients with poor breast aesthetic effect, 41.82% with an “excellent” rating, and 10% with a “good” and “fair” rating. After operation, the proportion of patients with an “excellent” rating was increased to about 71.29%, while the proportion of patients with a “poor” rating was reduced to less than 1%. And at 6 months after operation, all patients had excellent aesthetic evaluation results (Figure 2).

## 4. Discussion

Breast is an important sexual characteristic of women, but BC has a gradually rising incidence and poses a threat to patient health and even life. Surgery is an effective method for BC, which can improve the clinical symptoms of patients to a certain extent. However, surgical removal of the breast affects the appearance of patients, bringing psychological distress (such as depression, anxiety, and depressed mood) and leading to impaired quality of life [13]. In addition, the clinical detection rate and 5-year survival rate of BC are increasing [14]. Therefore, the quality of life of postoperative BC patients has become the focus of attention, and breast reconstruction is beginning to be favored.

Studies have reported that breast reconstruction has been considered as part of the treatment standard for patients undergoing mastectomy [15]. Breast reconstruction allows patients to restore their physical shape to a certain extent, thus reducing their psychological pressure, restoring self-confidence, and improving postoperative quality of life [16, 17]. There are two timings of breast reconstruction, IBR and DBR. In the early stage, DBR is mostly used for breast reconstruction due to a worry that IBR will increase the tumor recurrence rate, affect the effect of adjuvant therapy, and therefore reduce the quality of life of patients [18]. Additionally, the reconstructed breast cannot be comparable to the original one, and DBR can allow patients to adapt to and accept postoperative body shape changes [18]. However, in comparison with patients with IBR, patients with DBR are more likely to have problems in body image, emotion, and social stress, especially during the process of waiting for reconstruction [15]. And currently, there is no evidence that IBR increases the risk of postoperative recurrence and death [2]. A longitudinal study of 30 patients with IBR after BC surgery found that the quality of life was significantly improved at 12 months and 18 months after IBR, with significant differences in anxiety and depression compared with those before IBR [19]. IBR can avoid the psychological pressure during the time waiting for reconstruction and reduce the occurrence of negative emotions [19]. A study of 117 patients with IBR also pointed out that compared with simple mastectomy, IBR results in a lower incidence of anxiety and depression; and IBR is superior to DBR in terms of mental health, overall aesthetics, and cost-effectiveness [20]. Additionally, in a satisfaction study of patients receiving IBR, they stated that IBR has brought their physical appearance closer to normal, made them to be more confident in their bodies, and improved postoperative quality of life, thus allowing them to get rid of cancer and start a new life [21]. Howes et al. [22] showed that IBR after mastectomy significantly improved the postoperative cosmetic results without affecting the long-term efficacy, which could obtain better satisfaction and body image and ensure the postoperative quality of life. And IBR is able to reduce the occurrence of postoperative complications [23], while it does not increase local tumor recurrence and distant metastasis [24, 25]. In this study, it was found that IBR significantly improved the breast aesthetic effect, postoperative skin texture, appearance of the reconstructed breast, and nipple shape, with high safety. Our findings are consistent with previous study results. Because this study is a prospective multicenter observational study, it is not supported by experimental results of detection and has certain limitations. However, the preliminary study results of this study showed can still conclude that IBR can significantly improve the quality of life of patients, which has a promising application for the treatment of BC patients.

## 5. Conclusion

In summary, IBR after mastectomy not only remodels the patient's breast but also improves the postoperative quality of life. This operation takes into account the aesthetic effect, without increasing the occurrence of postoperative complications, with high safety. It is suggested that clinicians should make a correct preoperative decision on the premise of considering patients' survival status and postoperative quality of life, thus realizing accurate individualized treatment of BC.

## Figures and Tables

**Figure 1:** FACT-B scores of patients in the perioperative period and at 3 and 6 months after operation. ^*∗∗*^*P* < 0.01 vs. the perioperative period group.

**Figure 2:** Postoperative breast aesthetics in the perioperative period and at 3 and 6 months after operation.

**Table 1:** Clinical baseline characteristics of the patients.

Variables	Total *N* = 878	Mean ± SD/*n* (%)	Missing value
Age, years		46.28 ± 9.43	124.00
BMI (body mass index)		22.62 ± 3.87	1.00

Income			121.00
	<5000	294 (38.84)	
	5000–10000	352 (46.50)	
	>10000	111 (14.66)	

Marital status			9.00
	Divorced	16 (1.84)	
	Married	99 (11.39)	
	Unmarried	754 (86.77)	

Give birth or not	Yes	192 (21.87)	
Number of pregnancies		2.23 ± 1.18	545.00
Number of deliveries		1.29 ± 0.55	545.00
Lactation or not	Yes	357 (40.66)	
Duration of lactation (months)		9.66 ± 4.48	575.00
Menopause or not		104 (11.85)	
Hypertension		17 (3.33)	367.00
Diabetes		3 (0.59)	367.00

Tumor location	Upper-inner	74 (16.86)	439.00
	Lower-inner	21 (4.78)	
	Upper-outer	246 (56.04)	
	Lower-outer	53 (12.07)	
	Central area	45 (10.25)	

Tumor size (cm)		2.24 ± 1.64	470.00
TNM staging			718.00 (value missing and classification too fine for statistics)
Distant metastasis	No distant metastasis	402 (94.37)	452.00
	Distant metastasis	24 (5.63)	

Histopathological grade	Nonassessable	89 (24.52)	515.00
	Low	70 (19.28)	
	Medium	146 (40.22)	
	High	58 (15.98)	

Pathological diagnosis	Invasive carcinoma	333 (76.55)	443.00
	Carcinoma in situ	78 (17.93)	
	Others	24 (5.52)	

**Table 2:** Postoperative outcomes of the patients.

Variables	Total *N* = 878	Mean ± SD/*n* (%)	Missing value
Postoperative chemotherapy	Yes	211 (50.48)	460.00
Number of drainage tubes	1	5 (1.16)	446.00
	2	395 (91.44)	
	3	28 (6.48)	
	4	4 (0.93)	
Immediate breast reconstruction		865 (98.52)	
Psychological status of patients at admission	Any one or more of anxiety, irritability, and fear	318 (77.00)	465.00
	Normal	95 (23.00)	
Acceptance of physical changes at discharge	Acceptable	23 (4.89)	408.00
	Unacceptable	442 (94.04)	
	No cognition	5 (1.06)	
Total hospital stay		15.87 ± 6.42	574.00
Total cost		12823.13 ± 32735.83	153.00
Recurrences		4 (0.83)	397.00
Metastasis		8 (1.67)	398.00

**Table 3:** Postoperative safety assessment.

	One month after operation	Three months after operation	Six months after operation	12 months after operation
Edema of the affected limb	5	21	0	0
Capsule contracture	3	26	0	0
Infection	13	1	0	0
Calcifications around the prosthesis	6	27	1	0
Prosthetic dislocation (exposure)	3	6	0	0
Hematoma or seroma	6	1	0	0
Delayed wound healing	2	7	1	0
Breast atrophy and thoracic deformity	3	31	0	0
Chronic lymphadenopathy	5	21	0	0
Pain	3	6	1	0
Prosthetic ruptures	16	31	0	0

**Table 4:** Follow-up at 3, 6, and 12 months after operation.

		Three months after operation	Six months after operation	12 months after operation
Skin texture	High elasticity	9	1	0
	Medium elasticity	62	13	3
	Low elasticity	34	2	0
	No elasticity	5	0	0
Appearance of the reconstructed breast	Normal	63	2	0
	Too high	11	4	0
	Asymmetric	28	10	3
Nipple shape	Protruded and normal in size	77	10	3
	Inverted	9	2	0
	Ptosis	3	1	0

## Data Availability

The data used to support the findings of this study are available from the corresponding author (Chao Zhang) upon request.
